# Antisecretory and Spasmolytic Activities of Aqueous and Ethanolic Stem Bark Extracts of *Nauclea diderrichii* in Wistar Rats

**DOI:** 10.1155/2022/7569848

**Published:** 2022-06-19

**Authors:** R. C. Douho Djimeli, M. L. Nchouwet, S. L. Poualeu Kamani, L. M. Tchoumba Tchoumi, A. Kamanyi, S. L. Wansi Ngnokam

**Affiliations:** Laboratory of Animal Physiology and Phytopharmacology, Department of Animal Biology, Faculty of Sciences, University of Dschang, Cameroon

## Abstract

**Background:**

Diarrheal diseases are a major cause of morbidity and mortality throughout the world and particularly in developing countries. *Nauclea diderrichii* is a plant used in traditional medicine in the treatment of anemia, fever, gastric ulcer, malaria, abdominal pain, skin infections, and diarrhea. The present work is aimed at evaluating the antisecretory and spasmolytic activities of aqueous and ethanolic stem bark extracts of *Nauclea diderrichii* in Wistar rats.

**Methods:**

The effect of aqueous and ethanolic extracts of *Nauclea diderrichii* was tested at doses of 100, 200, and 300 mg/kg on castor oil-induced secretory diarrhea, misoprostol-induced fluid accumulation, and the effect of pretreatment with yohimbine and glibenclamide. They were also tested on normal motility and castor oil- and carbachol-induced hypermotility.

**Results:**

The results showed that the aqueous and ethanolic extracts of *Nauclea diderrichii* significantly (*p* < 0.001) inhibited castor oil-induced secretory diarrhea at all the doses. Both extracts significantly (*p* < 0.001) inhibit fluid accumulation induced by misoprostol. The pretreatment with glibenclamide reduced the antidiarrheal activity of aqueous extract of *Nauclea diderrichii*. The pretreatment with yohimbine did not alter the effect of the aqueous extract of *Nauclea diderrichii*. On intestine transit as on castor oil- and carbachol-induced motility, the aqueous and ethanolic extracts at doses of 100 and 200 mg/kg reduced significantly (*p* < 0.05, *p* < 0.01, and *p* < 0.001) the travelled distance by charcoal and peristaltic index.

**Conclusions:**

The study demonstrated that the aqueous and ethanolic extracts of *Nauclea diderrichii* possess antisecretory and antispasmolytic properties hence its use in traditional medicine against diarrhea.

## 1. Introduction

Diarrheal disease is the passage of 3 or more loose or liquid stools per day or more frequently than is normal for an individual [1]. It is usually a symptom of gastrointestinal infection, which can be caused by a variety of bacterial, viral, and parasitic organisms [1]. Diarrhea affects the gastrointestinal tract (GIT) and increases intestinal motility and secretory activities and decreases water and electrolyte absorption. The pathophysiological process of diarrhea includes increased intestinal osmolarity, excessive secretion of fluid and electrolytes, intestinal hypermotility, and a reduction in the absorptive processes and intestinal residence time [2].

Diarrheal diseases are the second leading cause of death in children under five years old and are responsible for killing around 525 000 children every year [1]. Diarrheal diseases are a major cause of morbidity and mortality throughout the world, particularly in developing countries [3].

Alternatively, many opioid drugs like diphenoxylate, loperamide, diloxanide furoate, racecadotril, and muscarinic receptor blockers like atropine sulfate are available in pharmacies for treating diarrhea. However, these synthetic substances are associated with adverse effects including vomiting, gastrointestinal discomfort, convulsion, constipation, and headache [4, 5]. Despite immense technological advancement in modern medicine and addition to adverse effects of synthetic substances, many developing countries still rely on healing practices and medicinal plants for their health care needs. A range of medicinal plants with antidiarrheal properties widely used by traditional medicines has not been scientifically evaluated [6]. Many studies have demonstrated the antidiarrheal properties of medicinal plants such as *Alchornea laxiflora* [7], *Distemonanthus benthamianus* [8], and *Mangifera indica* [9].

*Nauclea diderrichii* is a plant of the Rubiaceae family used folk in Cameroon in the treatment of anemia, fever, gastric ulcer, malaria, abdominal pain, skin infections, and diarrhea [10]. Scientific studies have shown that the extracts of this plant possess antiarthritic properties [11], antimalaria activities [12], and antileishmanian effects [13]. Phytochemical investigations have revealed the presence of phenols, triterpenes, sugars, alkaloids, tannins, glycosides, saponins, flavonoids, and cardiac glycosides [14, 15]. Tannins, alkaloids, flavonoids, and terpenoids are the major constituents that are primarily responsible for the antidiarrheal activity of medicinal plants [16]. Tannins are known to reduce secretion and make intestinal mucus resistant through the formation of protein tannate [17]. In view of all the above, we have undertaken this work with the aim of evaluating the antisecretory and spasmolytic activities of the aqueous and ethanolic extracts of the stem barks of *Nauclea diderrichii* in Wistar rats.

## 2. Materials and Methods

### 2.1. Drugs and Chemicals

Loperamide was obtained from Biotech Co., Ltd (Shaanxi, China); misoprostol (Cytotec) was purchased from Pfizer Holding, France. Activated charcoal (Carbophos E153) was obtained from Tradiphar (Lille, France); castor oil, distilled water, and ethanol were obtained from Geochim (Geochim, Cameroon). Atropine sulfate was obtained from Sigma Aldrich (St. Louis, MO63103, USA). Sodium chloride (NaCl), glibenclamide, and yohimbine were obtained from Sigma Chemicals Co., UK.

### 2.2. Plant Material and Extraction

*Nauclea diderrichii* stem bark was harvested at Mbanga (Moungo Division, Littoral region of Cameroon) in March 2019 and authentified at Cameroon National Herbarium (CNH) by comparison with the voucher specimen registered under the reference number 6608/HNC. *Nauclea diderrichii* stem bark was sliced, dried at room temperature (24-25°C), and ground to a fine powder which was used for aqueous and ethanolic extractions. The aqueous extract was prepared by boiling 500 g of powder in 5000 ml of distilled water for 20 minutes. The resulting mixture was filtered using Whatman paper no. 4. After filtration, the filtrate was dried in an oven at 40°C for 2 days. This process allowed 44.37 g of aqueous extract (AEND) for an extraction yield of 8.874%. Concerning ethanolic extract, 500 g of the same powder was macerated in 5000 ml of ethanol (96%) for 48 hours. The resulting mixture was filtered using Whatman paper no. 4, and filtrate was evaporated using a rotavapor under reduced pressure (79°C), giving 24.35 g of ethanolic extract (EEND) for an extraction yield of 4.87%.

### 2.3. Animals

Wistar rats of both sexes, age 8 to 10 weeks and weighing 90 to 120 g, were used. They were bred at the animal house of the Department of Animal Biology of the Faculty of Sciences of the University of Dschang under natural room conditions. Animals were fed a standard diet and received water ad libitum. Prior to the experimental protocol, the rats were acclimated for 48 hours to laboratory conditions with natural light (12 hours on natural light and 12 hours dark) for minimizing any nonspecific stress. Experimental protocols used in this study were approved by the laboratory committee Research Unit of Animal Physiology and Phytopharmacology, Department of Animal Biology, Faculty of Sciences, the University of Dschang-Cameroon) according to the standard ethical guidelines for laboratory use and care as described in the European Community guidelines, EEC directive 86/609/EEC, of the 24th of November 1986.

### 2.4. Evaluation of Antisecretory Activity of the Aqueous and Ethanolic Extracts of *Nauclea diderrichii*

#### 2.4.1. Castor Oil-Induced Secretory Diarrhea

Secretory diarrhea was induced following the modified protocol described by Karthik et al. [18] with slight modifications. Thus, sixty (60) rats were housed separately in wire-mesh cages and fasted for 24 hours. The filter paper was placed under each box to collect the feces. After 24 hours of observation, only animals who showed no signs of diarrhea were retained and randomly divided into ten groups of six animals each: group 1 served as neutral control and received distilled water (10 ml/kg *p.o.*); groups 2 and 3 served as negative control and received distilled water and DMSO (5%), respectively (10 ml/kg *p.o.*); group 4 served as positive control and was treated with loperamide at a dose of 2.5 mg/kg; groups 5, 6, and 7 were treated with AEND at the respective doses of 100, 200, and 300 mg/kg; and groups 8, 9, and 10 were treated with EEND at the respective doses of 100, 200, and 300 mg/kg. The animals retained for this test received the different doses of extracts as well as the reference substance orally at the volume of administration of 1 ml per 100 g of body weight. One hour after administration of the various treatments, the animals received orally castor oil at the rate of 1 ml per 100 g of body weight with the exception of group 1 animals which received distilled water.

The animals were observed for six hours postgavage, and the following parameters were evaluated: time of onset of diarrhea, the frequency of diarrheal stools, the total emission of stools, and stool water content. The percentage inhibition (%*I*) of diarrhea was calculated as follows:

(1) $$\begin{array}{c} \%\text{inhibition}=\frac{\left(\text{wet defecation}\right)\text{control}-\left(\text{wet defecation}\right)\text{test}}{\left(\text{wet defecation}\right)\text{control}}\times 100. \end{array}$$

#### 2.4.2. Misoprostol-Induced Fluid Accumulation

This experiment was carried out according to the protocol described by Wondmagegn et al. [19] with slight modifications. Thus, the rats were fasted for 24 hours and divided into 10 groups of 6 rats each. They were treated as follows: group 1 served as neutral control and received distilled water (10 ml/kg *p.o.*); groups 2 and 3 served as negative control and received distilled water and DMSO (5%), respectively (10 ml/kg *p.o.*); group 4 served as positive control and treated with loperamide at a dose of 2.5 mg/kg; groups 5, 6, and 7 were treated with AEND at the respective doses of 100, 200, and 300 mg/kg; and groups 8, 9, and 10 were treated with EEND at the respective doses of 100, 200, and 300 mg/kg. The animals retained for this test received the different doses of extracts as well as the reference substance orally at the volume of administration of 1 ml per 100 g of body weight. One hour after treatment, the rats received misoprostol orally at the volume of administration of 1 ml/100 g of body weight with the exception of group 1 animals which received distilled water.

After one hour, they were anesthetized by injection of 0.5 ml of ketamine (50 mg/kg) and 0.5 ml of diazepam (10 mg/kg). Then, the entire abdominal cavity was opened, and the section of the small intestine from the pyloric sphincter to the ileocoecal junction was removed, after placing tight ligature at the ends. The small intestine was removed, and the intestinal contents were collected in a graduated cylindrical tube to measure its volume. The antisecretory activity expressed as a percentage of inhibition (%*I*) was calculated as follows:

(2) $$\begin{array}{c} \%\text{inhibition}=\frac{\left(\text{intestinal volume}\right)\text{control}-\left(\text{intestinal volume}\right)\text{test}}{\left(\text{intestinal volume}\right)\text{control}}\times 100. \end{array}$$

The intestinal content was subsequently centrifuged at 3000 rpm for 15 minutes, and the supernatant was collected for the determination of K^+^, Na^+^, Ca^2+^, and Cl^−^ ion concentrations.

The concentration of the ions was determined by spectrophotometry using commercial kits.

#### 2.4.3. Effect of Yohimbine and Glibenclamide on Antidiarrheal Activity of Aqueous Extract

This experiment was carried out according to the protocol described by Noubissi [20]. Thus, the rats were fasted for 24 hours and divided into 8 groups of 6 rats each. They were treated as follows: group 1 served as neutral control and received distilled water (10 ml/kg *p.o.*), group 2 served as negative control and received distilled water (10 ml/kg *p.o.*), group 3 served as positive control and was treated with loperamide at a dose of 2.5 mg/kg, group 4 was treated with AEND 300, group 5 was treated with glibenclamide (1 mg/kg) and AEND 300, group 6 was treated with yohimbine (1 mg/kg) and AEND 300, group 7 was treated with glibenclamide (1 mg/kg), and group 8 was treated with yohimbine (1 mg/kg). The animals retained for this test received the different substances orally at the volume of administration of 1 ml per 100 g of body weight with the exception of the yohimbine which was administered by subcutaneous route. Thirty minutes after administration of the various treatments, the animals received orally castor oil at the rate of 1 ml per 100 g of body weight.

The animals were observed for six hours postgavage, and the following parameters were evaluated: time of onset of diarrhea, the frequency of diarrheal stools, the total emission of stools, and the stool water content. The percentage inhibition (%*I*) of diarrhea was calculated as follows:

(3) $$\begin{array}{c} \%\text{inhibition}=\frac{\left(\text{wet defecation}\right)\text{control}-\left(\text{wet defecation}\right)\text{test}}{\left(\text{wet defecation}\right)\text{control}}\times 100. \end{array}$$

### 2.5. Evaluation of Spasmolytic Activity of the Aqueous and Ethanolic Extracts of *Nauclea diderrichii*

#### 2.5.1. Normal Motility

The effect of the extracts on normal motility was investigated following the method described by Tadesse et al. [21] with slight modifications. Fifty-four (54) rats were individually separated in the boxes of the screened cage and fasted for 18 hours and divided into 9 groups of 6 rats each and treated by gavage as follows: groups 1 and 2 served as neutral control and received distilled water and DMSO (5%), respectively (10 ml/kg *p.o.*); group 3 served as positive control and was treated with atropine sulfate at a dose of 1 mg/kg; groups 4, 5, and 6 were treated with AEND at the respective doses of 100, 200, and 300 mg/kg; and groups 7, 8, and 9 were treated with EEND at the respective doses of 100, 200, and 300 mg/kg.

Sixty minutes after administration of these different treatments, each rat orally received 1 ml/100 g of deactivated charcoal (10%) (Tradiphar); 60 minutes after, they were sacrificed after injection of 0.5 ml of ketamine (50 mg/kg) and 0.5 ml of diazepam (10 mg/kg). Then, the section of the small intestine from the pylorus to the caecum was sampled and deployed, and the distance traveled by the coal was measured. The peristaltic index (PI) was calculated as follows:

(4) $$\begin{array}{c} \text{Peristaltic index }\left(\text{PI}\right)=\frac{\text{Distance traveled }}{\text{Intestine total length }}\times 100. \end{array}$$

The percentage inhibition (%*I*) was calculated as follows:

(5) $$\begin{array}{c} \%\text{inhibition}=\frac{\left(\text{PI}\right)\text{control}-\left(\text{PI}\right)\text{test}}{\left(\text{PI}\right)\text{control}}\times 100. \end{array}$$

#### 2.5.2. Castor Oil-Induced Transit Acceleration

The acceleration of intestinal transit induced by castor oil was done according to the method described by Tadesse et al. [21] with slight modification. Sixty (60) rats fasted for 24 hours and were divided into 10 groups of 6 rats each and treated by gavage as follows: group 1 served as neutral control and received distilled water (10 ml/kg, *p.o.*); groups 2 and 3 or negative control received, respectively, distilled water and a 5% DMSO (10 ml/kg, *p.o.*); group 4 or positive control received atropine sulfate at a dose of 1 mg/kg; groups 5, 6, and 7 were treated with AEND at doses of 100, 200, and 300 mg/kg, respectively; and groups 8, 9, and 10 were treated with EEND at doses of 100, 200, and 300 mg/kg, respectively. Sixty minutes after administration of these different treatments, each rat received orally 1 ml/100 g body weight of castor oil with the exception of group 1 animals which received distilled water; and 30 minutes after administration of castor oil, they received orally 1 ml/100 g body weight of deactivated charcoal (Tradiphar); 60 minutes after, they were sacrificed after injection of 0.5 ml of ketamine (50 mg/kg) and 0.5 ml of diazepam (10 mg/kg). Then, the section of the small intestine from the pylorus to the caecum was sampled and deployed, and the distance traveled by the coal was measured. The peristaltic index (PI) was calculated as follows:

(6) $$\begin{array}{c} \text{Peristaltic index }\left(\text{PI}\right)=\frac{\text{Distance traveled }}{\text{Intestine total length }}\times 100. \end{array}$$

The percentage inhibition (%*I*) was calculated as follows:

(7) $$\begin{array}{c} \%\text{inhibition}=\frac{\left(\text{PI }\right)\text{control}-\left(\text{PI }\right)\text{test}}{\left(\text{PI }\right)\text{control}}\times 100. \end{array}$$

#### 2.5.3. Carbachol-Induced Transit Acceleration

The acceleration of intestinal transit by carbachol was evaluated following the protocol described by Noubissi et al. [22]. Sixty (60) rats fasted for 18 hours and were divided into 10 groups of 6 rats each and treated as in the previous test. Thirty minutes after administration of the different treatments, carbachol hydrochloride (0.5 mg/kg) was administered intraperitoneally to the animals. Immediately after administration of carbachol, each animal received orally 1 ml/100 g bw of deactivated charcoal (Tradiphar) except for group 1 animals which received distilled water.

Sixty (60) minutes after, they were sacrificed after injection of 0.5 ml of ketamine (50 mg/kg) and 0.5 ml of diazepam (10 mg/kg). Then, the section of the small intestine from the pylorus to the caecum was sampled and deployed, and the distance traveled by the coal was measured. The peristaltic index (PI) was calculated as follows:

(8) $$\begin{array}{c} \text{Peristaltic index }\left(\text{PI}\right)=\frac{\text{Distance traveled }}{\text{Intestine total length }}\times 100. \end{array}$$

The percentage inhibition (%*I*) was calculated as follows:

(9) $$\begin{array}{c} \%\text{inhibition}=\frac{\left(\text{PI}\right)\text{control}-\left(\text{PI}\right)\text{test}}{\left(\text{PI}\right)\text{control}}\times 100. \end{array}$$

### 2.6. Statistical Analysis

Statistical analysis was performed using GraphPad Prism version 8.4.2 statistical software. The data obtained were expressed as the mean ± standard error on mean (SEM). All groups were compared using one-way analysis followed by the Tukey posttest. Differences were considered statistically significant at *p* < 0.05.

## 3. Results

### 3.1. Antisecretory Activities of Aqueous and Ethanolic Extracts of *Nauclea diderrichii*

#### 3.1.1. Effect of Aqueous and Ethanolic Extracts of *Nauclea diderrichii* on Secretory Diarrhea Induced by Castor Oil

Table 1 shows the antisecretory effect of the aqueous and ethanolic stem bark extract of *Nauclea diderrichii*. It follows that castor oil causes a significant (*p* < 0.001) reduction of the onset time and increases significantly (*p* < 0.001) the total stool frequency, diarrheal stool frequency, and water content of negative control in comparison with neutral control. The aqueous and ethanolic extracts of *Nauclea diderrichii* significantly (*p* < 0.001) increase the onset time at all the doses and significantly (*p* < 0.001) decrease the total stool frequency, diarrheal stool frequency, and water content in comparison with negative control. The best inhibition was obtained at a dose of 300 mg/kg with 93.40% of inhibition for aqueous extract and at the dose of 200 mg/kg with 82.23% of inhibition for ethanolic extracts. The activities of the extracts were similar to those of loperamide (2.5 mg/kg) which led to 100% of inhibition.

Each value represents the mean ± SEM (*n* = 6). ANOVA one way followed by Tukey's posttest. ^a^*p* < 0.05, ^b^*p* < 0.01, and ^c^*p* < 0.001: significant difference compared to the neutral control (distilled water (Neu)). ^∗^*p* < 0.05;  ^∗∗∗^*p* < 0.001: significant differences compared to the negative control (distilled water (Neg) or DMSO 5%.). DW: distilled water; Neu: neutral control; Neg: negative control; Lop: loperamide; Pos: positive control.

#### 3.1.2. Antiaccumulative Effect of the Aqueous and Ethanolic Stem Bark Extracts of *Nauclea diderrichii*

Table 2 shows the antiaccumulative effect of the aqueous and ethanolic stem bark extracts of *Nauclea diderrichii*. It follows that misoprostol causes a significant (*p* < 0.001) increase in volume of intestinal fluid and Na^+^, K^+^, Ca^2+^, and Cl^−^ concentration compared to neutral control. However, the administration of the aqueous and ethanolic extracts of *Nauclea diderrichii* significantly (*p* < 0.001) decreases the volume of intestinal fluid and Na^+^, K^+^, Ca^2+^, and Cl^−^ concentration compared to negative control. The best inhibition was obtained at a dose of 200 mg/kg of the ethanolic extract with 44.60% of inhibition. The activity of the extract was similar to those of loperamide (2.5 mg/kg) which led to 36.58% of inhibition.

Each value represents the mean ± SEM (*n* = 6). ANOVA one way followed by Tukey's posttest. ^b^*p* < 0.01; ^c^*p* < 0.001: significant difference compared to the neutral control (distilled water (Neu)). ^∗^*p* < 0.05,  ^∗∗^*p* < 0.01, and^∗∗∗^*p* < 0.001: significant difference compared to the negative control (distilled water (Neg) or DMSO 5% (Neg)). DW: distilled water; Neu: neutral control; Neg: negative control; Lop: loperamide; Pos: positive control.

#### 3.1.3. Effect of Pretreatment with Yohimbine and Glibenclamide on Antidiarrheal Activity of Aqueous Stem Bark Extract of *Nauclea diderichii*

Table 3 shows the effect of pretreatment with yohimbine and glibenclamide on antidiarrheal activity of the aqueous stem bark extract of *Nauclea diderichii*. The pretreatment of rats with glibenclamide significantly (*p* < 0.001) decreases antidiarrheal activity of the aqueous extract of *Nauclea diderrichii* (300 mg/kg). The aqueous extract alone inhibited diarrhea with 84.42% of inhibition, whereas the % of inhibition was 49.91 in animals pretreated with glibenclamide. The pretreatment of rats with yohimbine did not decrease antidiarrheal activity of the aqueous extract of *Nauclea diderrichii* (300 mg/kg). The aqueous extract alone inhibited diarrhea with 84.42% of inhibition, whereas the percentage of inhibition was 81.24% in animals pretreated with yohimbine.

Each value represents the mean ± SEM (*n* = 6). ANOVA one way followed by Tukey's posttest. ^b^*p* < 0.01; ^c^*p* < 0.001: significant difference compared to the neutral control (distilled water (Neu)). ^∗∗^*p* < 0.01;  ^∗∗∗^*p* < 0.001: significant difference compared to the negative control (distilled water (Neg)). DW: distilled water; Neu: neutral control; Neg: negative control; Lop: loperamide; Pos: positive control; GLIB: glibenclamide; YOHI: yohimbine; AE: aqueous extract of *Nauclea diderrichii*.

### 3.2. Evaluation of Spasmolytic Activity of the Aqueous and Ethanolic Extracts of *Nauclea diderrichii*

#### 3.2.1. Spasmolytic Effect of the Aqueous and Ethanolic Stem Bark Extracts of *Nauclea diderrichii* on Normal Intestinal Motility

The results summarised in Table 4 present the effect of the aqueous and ethanolic extracts of stem bark of *Nauclea diderrichii* on normal motility. It follows from the table that the two extracts reduce the charcoal propulsion with the best effect which is obtained at the doses of 300 and 200 mg/kg, respectively. At these doses, the aqueous and ethanolic extracts significantly (*p* < 0.05 and *p* < 0.01, respectively) reduce charcoal propulsion (58.00 ± 4.20 and 68.00 ± 7.05, respectively) which led to a significant (*p* < 0.05 and *p* < 0.01, respectively) peristaltic index (55.43 ± 5.01 and 61.80 ± 6.33, respectively) compared to neutral control. The highest inhibition of 32.70% is obtained with a dose of 200 mg/kg of ethanolic extract, which is closely similar to that of the reference drug atropine sulfate (31.08%).

Each value represents the mean ± SEM (*n* = 6). ANOVA one way followed by Tukey's posttest. ^b^*p* < 0.01; ^c^*p* < 0.001: significant difference compared to the neutral control (distilled water); ^∗^*p* < 0.05: significant difference compared to the neutral control (DMSO (5%)).

#### 3.2.2. Spasmolytic Effect of the Aqueous and Ethanolic Stem Bark Extracts of *Nauclea diderrichii* on Castor Oil-Induced Intestinal Motility

Table 5 shows that castor oil has increased the intestine propulsion of charcoal and peristaltic index in rats compared with neutral control. Atropine sulfate, AEND, and EEND significantly (*p* < 0.05, *p* < 0.01, and *p* < 0.001) inhibited castor oil-induced intestine transit with the best inhibition of 50.67% for atropine and 40.59% for EEND at the dose of 300 mg/kg.

Each value represents the mean ± SEM (*n* = 6). ANOVA one way followed by Tukey's posttest. ^a^*p* < 0.05,  ^b^*p* < 0.01, and^c^*p* < 0.001: significant difference compared to the neutral control (distilled water (Neu)); ^∗^*p* < 0.05: significant difference compared to the negative control (distilled water (Neg) or DMSO). DW: distilled water; Neu: neutral control; Neg: negative control.

#### 3.2.3. Spasmolytic Effect of the Aqueous and Ethanolic Stem Bark Extracts of *Nauclea diderrichii* on Carbachol-Induced Intestinal Motility

Table 6 shows that carbachol has increased the intestine propulsion of charcoal and peristaltic index in rats compared with neutral control. Atropine sulfate, AEND, and EEND significantly (*p* < 0.05, *p* < 0.01, and *p* < 0.001) inhibited carbachol-induced intestine transit with the best inhibition of 39.71% for atropine and 36.00% for AEND at the dose of 200 mg/kg.

Each value represents the mean ± SEM (*n* = 6). ANOVA one way followed by Tukey's posttest. ^a^*p* < 0.05,  ^b^*p* < 0.01, and^c^*p* < 0.001: significant difference compared to the neutral control (distilled water (Neu)); ^∗^*p* < 0.05: significant difference compared to the negative control (distilled water (Neg) or DMSO). DW: distilled water; Neu: neutral control; Neg: negative control.

## 4. Discussion

This study was designed to evaluate the antisecretory and spasmolytic activities of the aqueous and ethanolic extracts of stem barks of *Nauclea diderrichii* in rats. Secretory diarrhea is the most dangerous frequent form of gastrointestinal pathology [23, 24]. Castor oil-induced diarrhea is a model generally used to assess the antisecretory potential of pharmacological substances. Castor oil contains an active metabolite called ricinoleic acid which is released after digestion of this oil by lipases [25]. Ricinoleic acid causes irritation and inflammation of the intestinal mucosa, thus releasing endogenous prostaglandin type E_2_ (PGE_2_) which stimulates peristaltic activity and intestinal secretion [25]. Ricinoleic acid also stimulates epithelial cells to produce nitric oxide and adenylate cyclase that lead to the production of prostaglandin-induced diarrhea [26]. In this study, castor oil significantly (*p* < 0.001) reduces the onset time and significantly (*p* < 0.001) increases the total stool frequency, diarrheal stool frequency, and water content. The aqueous and ethanolic extracts of the stem bark of *Nauclea diderrichii* and loperamide significantly (*p* < 0.001) increase the onset time and significantly (*p* < 0.001) decrease total stool frequency, diarrheal stool frequency, and water content. It can therefore be assumed that the antidiarrheal activity of aqueous and ethanolic extract can be mediated by an antisecretory or spasmolytic mechanism. This was evident from the decrease in the total number of wet feces in the test group [27]. Loperamide used as a reference substance is an opioid *μ*-receptor agonist that increases absorption and/or decreases gastrointestinal secretion or motility by activating *μ*-receptors in the myenteric plexus of the large intestine [28, 29]. Activation of these receptors inhibits the release of acetylcholine resulting in relaxation of the intestinal smooth muscle [30]. The aqueous and ethanolic extracts of *Nauclea diderrichii* would therefore be capable of interfering either with the production or action of prostaglandin E_2_ or with the acetylcholine mechanism because they have similar activities to loperamide.

To elucidate the mechanism of action, the antiaccumulation was also tested using a misoprostol-induced enteropooling assay in rats. Misoprostol is a synthetic analogue of PGE_2_ which generates an accumulation of intestinal fluid and stimulates the secretion of mucus [31]. The administration of misoprostol significantly (*p* < 0.001) increases the volume of intestinal fluid and the intestinal concentration of Na^+^, K^+^, Ca^2+^, and Cl^−^. The aqueous and ethanolic extracts of *Nauclea diderrichii* significantly (*p* < 0.001) reduce the volume of the fluid intestine and the intestinal concentration of Na^+^, K^+^, Ca^2+^, and Cl^−^. These results suggest that the aqueous extract contains a substance that is able to inhibit the prostaglandin biosynthesis or block prostaglandin receptors.

Glibenclamide is a potassium receptor antagonist, and when it binds to potassium receptors, it blocks potassium channels resulting in the depolarisation of intestinal smooth muscle cells with the opening of voltage-dependent calcium channels and entry of calcium [32]. On the other hand, its opening leads to the entry of K^+^ ions followed by hyperpolarisation and thus the closing of voltage-dependent calcium channels, and thus, the consequence is muscle relaxation [32]. In this study, glibenclamide reduced the antidiarrheal activity of AEND, suggesting that glibenclamide lifted the inhibition caused by AEND and showing that AEND would act by activating the opening of potassium channels. This would be due to the presence in the extracts of flavonoids that have this ability to activate the opening of KATP channels [33]. Yohimbine is an *α*2-adrenergic receptor antagonist; by binding to these receptors, it decreases the absorption of fluids and electrolytes [32]. Pretreatment with yohimbine did not alter the effect of the aqueous extract of *Nauclea diderrichii*. This suggests that the action of aqueous extract of *Nauclea diderrichii* does not involve the *α*2-adrenergic receptor pathway.

Increasing intestinal motility is one way of increasing the formation of diarrhea. Ricinoleic acid is capable of increasing the peristalsis which leads to diarrhea [34]. In this study, the aqueous and ethanolic extracts of *Nauclea diderrichii* show a spasmolytic activity in the normal transit and on castor oil-induced hypermotility. The atropine sulfate used in this test as a reference substance is an antimuscarinic agent because it suppresses the movement of charcoal through its anticholinergic effect, and it acts as a cholinergic antagonist by binding to acetylcholine muscarinic receptors in the central and peripheral nervous systems [35]. The results obtained with the aqueous and ethanolic extracts show that these extracts would have acted by a mechanism similar to that of atropine sulfate.

To elucidate the mechanism of action, the effect of the extracts was tested on carbachol-induced intestinal transit. Carbachol is an agonist of M_3_ receptors of acetylcholine. Acetylcholine release as the major neurotransmitter from the autonomic nervous system (ANS) stimulates the intestinal smooth muscle due to muscarinic receptor action [36]. The activation of the muscarinic receptor specifically M_3_ subtype by acetylcholine stimulates phospholipase C (PLC) that subsequently caused the production of diacylglycerol (DAG) and inositol triphosphate (IP_3_). The IP_3_ stimulates the intracellular calcium ion (Ca^2+^) and mobilizes the release of Ca^2+^ from other tissues via a Ca^2+^-sensitive channel. The DAG phosphorylates the different proteins by stimulating the protein kinase C which subsequently activates the nonselective cationic channel and stimulated the voltage-dependent calcium channel [37]. Glibenclamide is a potassium channel antagonist; by binding to potassium channels, it causes depolarisation of intestinal smooth muscle cells with the opening of voltage-dependent calcium channels and entry of calcium [32]. The opening of potassium channels leads to the entry of K^+^ ions followed by hyperpolarisation [32]. The administration of carbachol increases intestine propulsion charcoal and peristaltic index. The aqueous and ethanolic extracts decrease intestine propulsion charcoal and peristaltic index. These results suggest that the extracts of *Nauclea diderrichii*, like atropine sulfate, which is a muscarinic antagonist of the M_3_ acetylcholine receptors, are said to contain substances that prevent the mobilization of intracellular calcium at the origin of muscular contraction; they also contain substances that block the M_3_ muscarinic receptors.

Phytochemical investigations on extracts of *Nauclea diderrichii* have revealed the presence of phenols, triterpenes, sugars, alkaloids, tannins, glycosides, saponins, flavonoids, and cardiac glycosides [14, 15]. Tannins reduce the intracellular Ca^2+^ inward current by stimulating the calcium channel, which induces muscle relaxation, ascribed to their spasmolytic and calcium channel blocking activities resulting in inhibition of intestinal peristaltic [7, 38]. Tannins are known to reduce secretion and make intestinal mucus resistant through the formation of protein tannate [17]. Flavonoids are known to have an antimotility mechanism through relaxing intestinal muscle [39, 40]. The aqueous and ethanolic extracts of *Nauclea diderrichii* possess antisecretory and spasmolytic activities due to the secondary metabolites present in the extracts.

## 5. Conclusions

The finding of the present study demonstrated that the aqueous and ethanolic extracts of *Nauclea diderrichii* are endowed with antidiarrheal activities. This antidiarrheal activity is due to the antisecretory and spasmolytic mechanism. The antisecretory and spasmolytic mechanism may be attributed to the presence of secondary metabolites in the extracts including flavonoids, tannins, triterpenes, saponins, phenols, and alkaloids. These effects justified the use of the plant as a nonspecific antidiarrheal agent in traditional medicine.

## Figures and Tables

**Table 1:** Antisecretory effects of aqueous and ethanolic extracts of *Nauclea diderrichii* on castor oil-induced diarrhea.

Treatments	Doses (mg/kg)	Onset time (min)	Total stool frequency	Diarrheal stool frequency	Inhibition (%)	Water content (%)
DW (Neu)	1 ml/100 g	360.00 ± 0.00	0.00 ± 0.00	0.00 ± 0.00	—	00.00 ± 00.00
DW (Neg)	1 ml/100 g	45.00 ± 3.31^c^	5.33 ± 0.21^c^	5.00 ± 0.63^c^	—	80.30 ± 0.85^c^
DMSO 5% (Neg)	1 ml/100 g	52.17 ± 4.20^c^	5.33 ± 0.21^c^	4.67 ± 0.33^c^	—	77.35 ± 2.89^c^
Lop (Pos)	2.5	360.00 ± 0.00^∗∗∗^	0.00 ± 0.00^∗∗∗^	0.00 ± 0.00^∗∗∗^	100	0.00 ± 0.00^∗∗∗^
Aqueous extract	100	72.67 ± 2.51^c∗∗∗^	1.83 ± 0.16^c∗∗∗^	1.50 ± 0.22^a∗∗∗^	70	58.76 ± 3.89^c^
	200	212.50 ± 14.83^c∗∗∗^	1.66 ± 0.21^c∗∗∗^	1.16 ± 0.16^∗∗∗^	76.80	69.25 ± 4.69^c^
	300	321.80 ± 9.00^a∗∗∗^	0.83 ± 0.16^b∗∗∗^	0.33 ± 0.21^∗∗∗^	93.40	56.54 ± 12.04^c∗^
Ethanolic extract	100	50.83 ± 9.09^c^	1.83 ± 0.17^c∗∗∗^	1.00 ± 0.26^b∗∗∗^	78.59	77.52 ± 3.36^c^
	200	91.33 ± 3.93^c∗^	1.33 ± 0.21^c∗∗∗^	0.83 ± 0.17^a∗∗∗^	82.23	67.28 ± 2.59^c∗^
	300	199.00 ± 15.06^c∗∗∗^	1.00 ± 0.00^c∗∗∗^	1.00 ± 0.00^b∗∗∗^	78.59	58.75 ± 4.37^c∗∗∗^

**Table 2:** Antiaccumulative effects of aqueous and ethanolic extracts of *Nauclea diderrichii* on misoprostol-induced enteropooling.

Treatments	Doses (mg/kg)	Volume of fluid (ml)	Na^+^ (mg/l)	K^+^ (mg/l)	Cl^−^ (mg/l)	Ca^2+^ (mg/l)
DW (Neu)	10 ml/kg	1.17 ± 0.08	22.41 ± 2.36	2.60 ± 0.02	2.11 ± 0.04	22.66 ± 1.96
DW (Neg)	10 ml/kg	2.05 ± 0.05^c^	53.20 ± 4.61^c^	5.07 ± 0.30^c^	4.13 ± 0.33^c^	49.35 ± 3.41^c^
DMSO 5% (Neg)	10 ml/kg	2.13 ± 0.08^c^	41.16 ± 1.34^c^	4.52 ± 0.13^c^	4.30 ± 0.29^c^	49.69 ± 2.69^c^
Lop (Pos)	2.5	1.30 ± 0.07^∗∗∗^	16.11 ± 1.50^∗∗∗^	2.59 ± 0.17^c∗∗∗^	1.71 ± 0.20^∗∗∗^	29.70 ± 3.85^∗∗∗^
Aqueous extract	100	1.17 ± 0.05^∗∗∗^	27.62 ± 2.05^∗∗∗^	5.17 ± 0.10^c^	2.18 ± 0.33^∗∗∗^	23.94 ± 3.57^∗∗∗^
	200	1.25 ± 0.05^∗∗∗^	52.08 ± 0.76	4.14 ± 0.21^c∗^	1.78 ± 0.12^∗∗∗^	33.43 ± 1.28^∗∗^
	300	1.20 ± 0.07^∗∗∗^	21.48 ± 1.53^∗∗∗^	3.93 ± 0.20^c∗∗^	1.61 ± 0.29^∗∗∗^	19.28 ± 2.04^∗∗∗^
Ethanolic extract	100	1.37 ± 0.08^∗∗∗^	17.78 ± 1.36^∗∗∗^	4.77 ± 0.15^c^	0.91 ± 0.33^b∗∗∗^	27.46 ± 5.27^∗∗∗^
	200	1.18 ± 0.12^∗∗∗^	10.73 ± 1.09^b∗∗∗^	3.12 ± 0.09^∗∗∗^	0.44 ± 0.12^c∗∗∗^	7.32 ± 1.79^∗∗∗^
	300	1.32 ± 0.09^∗∗∗^	21.34 ± 3.67^∗∗∗^	1.81 ± 0.06^c∗∗∗^	1.29 ± 0.04^a∗∗∗^	15.12 ± 32^∗∗∗^

**Table 3:** Effect of yohimbine and glibenclamide on antidiarrheal activity of aqueous extract of *Nauclea diderrichii* on castor oil-induced secretory diarrhea.

Treatments	Onset (min)	Total stool frequency	Diarrheal stool frequency	Inhibition (%)
DW (Neu)	360.00 ± 0.00	0.00 ± 0.00	0.00 ± 0.00	—
DW (Neg)	45.00 ± 3.31^c^	5.33 ± 0.21^c^	5.33 ± 0.21^c^	—
Lop (Pos)	360.00 ± 0.00^∗∗∗^	0.00 ± 0.00^∗∗∗^	0.00 ± 0.00^∗∗∗^	100
AE 300	321.80 ± 9.00^b∗∗∗^	0.83 ± 0.16^∗∗∗^	0.83 ± 0.16^∗∗∗^	84.42
GLIB (1 mg/kg)+AE 300	154.70 ± 9.44^c∗∗∗^	2.67 ± 0.33^c∗∗∗^	2.67 ± 0.33^c∗∗∗^	49.91
YOHI (1 mg/kg)+AE 300	314.70 ± 12.56^b∗∗∗^	1.00 ± 0.00^a∗∗∗^	1.00 ± 0.00^a∗∗∗^	81.24
GLIB (1 mg/kg)	93.50 ± 5.65^c∗∗∗^	4.33 ± 0.33^c^	4.33 ± 0.33^c^	18.76
YOHI (1 mg/kg)	107.50 ± 6.83^c∗∗∗^	3.83 ± 0.31^c∗∗^	3.83 ± 0.31^c∗∗^	28.14

**Table 4:** Spasmolytic effect of aqueous and ethanolic stem bark extracts of *Nauclea diderrichii* on normal motility.

Treatments	Dose (mg/kg)	Total length of intestine (cm)	Traveled distance by charcoal (cm)	Peristaltic index (%)	% inhibition
Distilled water	1 ml/100 g	107.20 ± 1.33	87.17 ± 5.82	81.13 ± 4.71	—
DMSO (5%)	1 ml/100 g	107.30 ± 3.52	98.83 ± 5.35	91.83 ± 2.92	—
Atropine sulfate	1	108.00 ± 2.66	59.83 ± 5.75^c∗^	55.91 ± 5.92^c∗^	31.08
Aqueous extract	100	107.00 ± 1.77	76.83 ± 7.29	71.44 ± 5.83	11.94
	200	107.30 ± 2.25	60.50 ± 7.05^∗^	55.92 ± 5.61^∗^	31.07
	300	105.30 ± 2.47	58.00 ± 4.20^∗^	55.43 ± 5.01^∗^	31.67
Ethanolic extract	100	106.80 ± 1.83	74.33 ± 2.32	69.50 ± 1.14^a^	24.32
	200	110.30 ± 4.18	68.00 ± 7.05^b^	61.80 ± 6.33^b^	32.70
	300	107.00 ± 1.61	72.33 ± 2.44^a^	67.58 ± 1.87^a^	26.40

**Table 5:** Effects of aqueous and ethanolic stem bark extracts of *Nauclea diderrichii* on castor oil-induced motility.

Treatments	Dose (mg/kg)	Total length of intestine (cm)	Traveled distance by charcoal (cm)	Peristaltic index (%)	% inhibition
DW (Neu)	1 ml/100 g	98.17 ± 1.08	75.33 ± 2.44	76.70 ± 2.03	—
DW (Neg)	1 ml/100 g	107.70 ± 3.68	81.83 ± 3.69	76.32 ± 3.87	—
DMSO (Neg)	1 ml/100 g	104.20 ± 1.70	80.67 ± 4.30	77.31 ± 3.42	—
Atropine	1	110.80 ± 1.17	41.67 ± 9.91^b∗∗∗^	37.65 ± 9.07^c∗∗∗^	50.67
Aqueous extract	100	107.20 ± 2.06	57.83 ± 4.50	54.17 ± 4.49	29.02
	200	106.20 ± 1.14	53.83 ± 6.47^∗^	50.71 ± 6.05^∗^	33.56
	300	106.80 ± 3.55	55.67 ± 4.22^∗^	52.46 ± 4.58^∗^	31.26
Ethanolic extract	100	105.20 ± 2.24	51.33 ± 3.85^a∗∗^	48.66 ± 3.18^b∗∗^	37.06
	200	107.50 ± 1.28	51.50 ± 1.54^a∗∗^	47.98 ± 1.73^b∗∗^	37.94
	300	105.50 ± 1.65	48.67 ± 5.29^a∗∗^	45.93 ± 4.74^c∗∗∗^	40.59

**Table 6:** Effects of aqueous and ethanolic stem bark extracts of *Nauclea diderichii* on carbachol-induced intestinal motility.

Treatments	Dose (mg/kg)	Total length of intestine (cm)	Traveled distance by charcoal (cm)	Peristaltic index (%)	% inhibition
DW (Neu)	1 ml/100 g	98.17 ± 1.08	75.33 ± 2.44	76.70 ± 2.03	—
DW (Neg)	1 ml/100 g	108.50 ± 2.29	103.80 ± 1.19	95.85 ± 1.62	—
DMSO (Neg)	1 ml/100 g	109.50 ± 1.38	105.80 ± 5.38	96.60 ± 1.23	—
Atropine	1	111.70 ± 1.80	64.50 ± 2.94^c∗^	57.79 ± 2.53^c∗^	39.71
Aqueous extract	100	107.80 ± 1.19	80.50 ± 2.04	74.78 ± 2.58	21.98
	200	111.50 ± 2.43	68.33 ± 1.11^∗^	61.34 ± 0.82^∗^	36.00
	300	103.20 ± 3.48	64.50 ± 2.99^∗^	62.38 ± 1.17^∗^	34.92
Ethanolic extract	100	110.80 ± 2.65	73.83 ± 1.49	66.80 ± 2.02^a^	30.85
	200	105.30 ± 3.48	75.33 ± 1.90^b^	71.70 ± 1.60^b^	27.78
	300	102.20 ± 3.71	68.33 ± 3.23^a^	66.82 ± 1.41^a^	30.82

## Data Availability

The data that support the findings of this study are available from corresponding author upon request.
